# Impact of Kangaroo Mother Care Intervention on Immunological and Pulmonary Functions of Preterm Infants during Breastfeeding

This article has been retracted.

**DOI:** 10.1155/2022/3180871

**Published:** 2022-05-19

**Authors:** Juan Yang, Yanan Guo, Yuying Dai

**Affiliations:** ^1^Department of Children Health Care & Breast-feeding, The Fourth Hospital of Shijiazhuang City, Shijiazhuang, China; ^2^Department of Pathogenic Biology, Chongqing Medical University, Chongqing, China; ^3^Obstetrics Department, Wei County Hospital of Traditional Chinese Medicine, Kaifeng, China

## Abstract

**Objective:**

Preterm infants (PTIs) are prone to respiratory failure or other diseases due to immature organ development and poor immunological function. Herein, the effects of Kangaroo Mother Care (KMC) on the immunological and pulmonary functions of PTIs during breastfeeding were investigated in this study.

**Methods:**

The study recruited 86 delivery women and their PTIs with preterm pregnancy outcomes, consisting of 46 cases receiving breastfeeding plus KMC intervention (KMC group) and 40 cases receiving breastfeeding plus routine care (control group). The time of first lactation, time of first breastfeeding, and duration of first breastfeeding were observed in both cohorts. The breastfeeding status was assessed using the LATCH system. Maternal psychological status was evaluated by the breastfeeding self-efficacy scale (BSES) and self-rating anxiety/depression scale (SAS/SDS). The growth and development of PTIs were recorded, and the levels of postalbumin (PA), transferrin (TRF), plasma albumin (ALB), immunoglobulin (Ig) *A*, Ig*G*, Ig*M*, and complement C3 and C4 were measured. The tidal volume (VT), tidal volume per kilogram (VT/kg), minute volume (MV), and minute volume per kilogram (MV/kg) were detected using a pulmonary function tester.

**Results:**

The KMC group presented shorter time of first lactation and first breastfeeding than the control group, with longer duration of first breastfeeding (*P* < 0.05). After intervention, the BSES scores of delivery women were increased, while the SAS and SDS scores were decreased, with more notable improvements in the KMC group (*P* < 0.05). The levels of PA, TRF, ALB, Ig*A*, Ig*G*, VT, and MV were elevated in PTIs in both groups, with more evident increase in the KMC group than in the control group (*P* < 0.05). A better growth of PTIs was found in the KMC group than the control group (*P* < 0.05).

**Conclusions:**

The study demonstrated that KMC intervention during breastfeeding could benefit PTIs specifically regarding their immunological and pulmonary functions.

## 1. Introduction

Unlike normal infants, preterm infants (PTIs) have a shorter gestational age, lower weight, and immature organ development, which predispose them to be complicated with other diseases, threatening the healthy development of newborns [1]. With the change of policies as well as some incentives such as the increase of elderly pregnant women and pregnancy complications in recent years, the premature birth rate has gradually increased, accounting for 5%–15% of the total number of deliveries [2]. Some premature babies have a good prognosis after positive treatment, while some others have adverse outcomes due to various diseases or improper nursing, which is an important factor causing premature infant death [3]. According to statistics, the global mortality rate of PTIs has reached 20.8%, showing an increasing trend [4]. PTIs with very low birthweight have an increased risk of abnormal lung function, particularly obstructive type and thoracic musculoskeletal abnormalities, which were related with alternations in lung function [5]. Additionally, PTIs born before 32 weeks' gestational age have high rates of late onset sepsis and necrotizing enterocolitis, which may be associated with both the infant's immune system and the developing gut microbiota [6].

Breast milk, the best natural nutritional supplement for newborns and the first choice for clinical treatment of PTIs, is of great significance to increase neonatal immunity and promote neonatal growth and development [7]. However, due to the poor condition of the child, pregnant women tend to develop anxiety and other negative emotions after delivery, which directly affects the maternal lactation function, leading to the reduction of the success rate of breastfeeding [8]. As the research deepens, the combination of effective interventions on the basis of conventional treatment has been found to exert a positive impact on the health level of delivery women and newborns. Kangaroo Mother Care (KMC), a way to imitate the animal kangaroo to take care of children, allows the delivery women to get in close contact with their infants as early as possible to shorten the interdependent relationship between them, which is extremely suitable for PTIs. At present, it has been fully put into clinical use in many countries with excellent application results [9, 10]. However, the research on KMC is in the theoretical guidance stage in China due to study on starting late, and there is still no comprehensive and abundant experimental evidence on the specific function improvement of KMC in PTIs, resulting in it not being widely used in clinical practice. Based on this, this study studies the improvement effect of KMC on the immunological function and pulmonary function of PTIs under breastfeeding, laying a reliable foundation for future application of KMC.

## 2. Methods

### 2.1. Enrollment of Study Subjects

After being reviewed and approval by the Ethics Committee of our hospital, 86 cases of delivery women and their PTIs with premature pregnancy outcomes in our hospital from March 2019 to August 2021 were selected for the study. Among them, 46 cases receiving KMC intervention during breastfeeding were assigned to the KMC group and 40 cases receiving routine intervention during breastfeeding were assigned to the control group. We obtained informed consent from all family members. Included PTIs must fulfill the following criteria: (i) gestational age of 28 to 37 weeks; (ii) birth weight <2500 g; (iii) head circumference <33 cm [11]; (iv) a singleton birth; and (v) vaginal delivery. PTIs were excluded out of the study if PTIs were diagnosed with cardiovascular diseases, blood system diseases, respiratory diseases, serious malformations, grade IV neonatal intraventricular hemorrhage, serious infectious diseases, genetic diseases, or congenital diseases; the delivery women had no ability to breastfeed; the delivery women had metabolic diseases; PTIs or the delivery women failed to complete treatment procedures for various reasons.

### 2.2. Treatment Protocols

The mother and baby assigned into the KMC group were arranged to meet in a clean indoor environment with appropriate temperature within two hours after delivery. Before the meeting, the medical staff including an attending doctor and two nurses carefully informed the mother about the posture of hugging the baby and the precautions for touching the baby. In the maternal semi-recumbent position, the child was placed naked between the mother's bare breasts. The mother placed one hand on the patient's back covered with a clean thin back, and the other hand supported the patient's buttocks to prevent the patient from sliding down. In this way, the child can fully feel the mother's smell and body temperature, thereby enhancing the emotional communication between the mother and the child, and stimulating the maternal lactation function. In addition, the medical staff paid close attention to the vital signs of the child, corrected the mother's practice in a timely manner, and encouraged the mother to communicate with the child softly. Finally, under the guidance of medical staff, the infant was helped to suck as early as possible. The initial KMC intervention lasted for half an hour, followed by two periods of 2 h at noon (generally 9:00–11:00) and 2 h in the afternoon (14:00–16:00). In the case of blood collection of children, the duration of KMC intervention was extended. The sucking reflex was established as early as possible, and the child's health was gradually restored. The control group: after birth, the nursing staff carried out airway cleaning, body cleansing, infection prevention, and measurement of body length, weight, and head circumference for the baby. The PTIs were placed in incubators at 32–34°C for real-time monitoring of vital signs. As for the mothers, health education and psychological counseling were provided so that they could understand the importance of breastfeeding until they could breastfeed. The treatment lasted for two weeks in both cohorts.

### 2.3. Detection Methods

The venous blood (3 mL) was extracted from included PTIs before and after intervention for the measurement of albumin (PA), transferrin (TRF), plasma albumin (ALB), immunoglobulin (Ig) *A*, Ig*G*, Ig*M*, and complement C3 and C4 levels with the use of an automatic biochemical analyzer. Besides, the tidal volume (VT), tidal volume per kilogram (VT/kg), minute volume (MV), and minute volume per kilogram (MV/kg) were detected using a pulmonary function tester.

### 2.4. Primary Outcomes

The breastfeeding status of PTIs was evaluated by the time of first lactation and first breastfeeding, as well as the duration of first breastfeeding. The maternal breastfeeding status was evaluated using the Latch, Audible swallowing, nipple Type, Comfort, Hold Scale (LATCH) system (the higher the score, the better the breastfeeding) [12]. The maternal confidence in breastfeeding was assessed using the breastfeeding self-efficacy scale (BSES), with higher scores representing higher confidence in breastfeeding [13]. The self-rating anxiety/depression scale (SAS/SDS) [14] were utilized to evaluate maternal psychological state (the higher the score, the worse the psychological state). The nutritional status of PTIs was assessed by detecting levels of postalbumin (PA), transferrin (TRF), and plasma albumin (ALB). The growth and development of PTIs were evaluated by weight increase, body length, head circumference, and upper arm circumference, with the growth efficiency calculated. The immunological function of PTIs was reflected by levels of Ig*A*, Ig*M*, and complement C3 and C4. The pulmonary function of PTIs was reflected by VT, VT/kg, MV, and MV/kg. When the delivery women were discharged from the hospital, they were given anonymous nursing satisfaction surveys to show their nursing satisfaction. The survey was conducted on a 10-point scale, with 10 being very satisfied, 7–9 being basically satisfied, 4–6 being improvement needed, and 1–3 being dissatisfied [15].

### 2.5. Statistics Processing

Data processing was made by SPSS23.0 (IBM, USA). Count data (expressed as percentage) were analyzed by Chi-square test. Measurement data (expressed as mean ± standard deviation) were tested by either paired or unpaired *t*-test. Statistical significance was assumed at *P* < 0.05.

## 3. Results

### 3.1. Baseline Data of Delivery Women and Their PTIs

Demographic and clinical data of two groups of delivery women and their PTIs were compared with regard to maternal age and BMI, gender distribution of newborn, gestational age, weight at birth, primiparity, and nationality. It was found that the KMC and control groups showed no significant difference in terms of maternal age and BMI, gender distribution of newborn, gestational age, weight at birth, the proportion of primiparity, and nationality (*P* > 0.05, Table 1).

### 3.2. KMC Intervention Benefited Breastfeeding Status of PTIs

The first lactation and first breastfeeding time in the KMC group were (39.14 ± 3.97 h) and (38.89 ± 4.16 h), respectively, which were lower than those in the control group (*P* < 0.05). A longer duration of first breastfeeding (12.87 ± 2.46 min) was observed in the KMC group versus the control group (6.08 ± 1.02) (*P* < 0.05). Besides, a higher LATCH score was found in the KMC group (7.07 ± 0.98) when comparable to the control group (6.25 ± 1.77) (*P* < 0.05, Table 2).

### 3.3. A Better Maternal Psychological State after KMC

Before receiving intervention, the BSES, SAS, and SDS scores showed no significant difference between the KMC group and the control group (*P* > 0.05). After intervention, the BSES scores were increased while the SAS and SDS scores were decreased in both groups (*P* < 0.05), with more significant changes in the KMC group in comparison with the control group (*P* < 0.05, Table 3).

### 3.4. Improved Nutrition and Growth of PTIs after KMC

The serum levels of PA, TRF, and ALB presented no distinct differences between the KMC group and the control group before intervention (*P* > 0.05), but all elevated significantly after intervention (*P* < 0.05). This elevation was more significant in the KMC group than the control group (*P* < 0.05, Figure 1). In comparison with the control group, the KMC group presented a better growth status, showing in weight gain, body length gain, head circumference increase, and upper arm circumference increase (*P* < 0.05, Table 4).

### 3.5. KMC Intervention Benefited Immunological and Pulmonary Functions of PTIs

It was found that the levels of Ig*A*, Ig*G*, Ig*M*, C3, and C4 exhibited no notable differences between the KMC group and the control group before intervention (*P* > 0.05), but all increased notably after intervention (*P* < 0.05), with higher levels in the KMC group as compared to the control group (*P* < 0.05, Figure 2). Similarly, the VT, VT/kg, MV, and MV/kg of PTIs in the KMC group and the control group had no statistical difference before receiving any intervention (*P* > 0.05). Two interventions improved the immunological and pulmonary functions of PTIs, but KMC improved more significantly (*P* < 0.05, Table 5).

### 3.6. A Better Maternal Satisfaction from KMC Intervention

The results of nursing satisfaction survey analysis showed none of included delivery women reporting being dissatisfied or improvement needed in the KMC group, with no evident difference between groups in terms of the number of cases rated dissatisfied or improvement needed (*P* > 0.05), while more cases in the KMC group were very satisfied with the intervention, with a statistical difference between the two groups (*P* < 0.05, Table 6).

## 4. Discussion

In recent years, PTIs have been more and more frequently seen in clinic. As their adaptability and organ function are not as good as those of term infants, the risk of organ dysfunction and infection as well as death after childbirth is significantly increased [16]. For PTIs, taking more targeted postpartum intervention measures is the key to ensuring their normal growth. Breastfeeding, as the best natural nutritional supplement, is of great significance to newborns. However, due to the organism particularity of PTIs, the contact between PTIs and their mothers is limited, which limits the effective implementation of breastfeeding [17]. And as premature mothers have just completed pregnancy, there are generally varying degrees of anxiety, depression, and other adverse psychology, which also greatly interferes with the output of breast milk [18]. Based on the above reasons, it is crucial to find an effective intervention for the development of newborns. By exploring the effect of KMC under breastfeeding, this study has important reference significance for clinical practice.

In this experiment, we first compared breastfeeding status between the two cohorts. The data revealed notably shorter time of first lactation and breast feeding in the KMC group, and higher duration of first breastfeeding, indicating that KMC can effectively promote maternal breast milk secretion after delivery and improve the efficiency of breastfeeding. The core of traditional intervention for PTIs is health education and life guidance, ignoring the importance of mother-infant contact and joint care [19], while the core concept of KMC, also known as skin contact care, is to enhance the direct contact between the mother and the baby, providing a warm environment similar to the womb for the newborn [20]. This change is bidirectional for mothers and babies. On the one hand, it can promote the growth and development of newborns by creating a good development environment for them. On the other hand, it can improve maternal happiness and the sense of achievement and relieve bad emotions [21]. As pointed out by Charpak N et al., KMC can effectively enhance the interaction between mother and baby, stimulate neurohypophysis and adenohypophysis, promote milk secretion, and release the emotion after childbirth by placing the newborn on the maternal chest and holding the newborn back with both hands [22]. This was also confirmed in the results of our survey on maternal breastfeeding confidence, and SAS and SDS scores, illustrating the positive effect of KMC on breastfeeding.

Second, ensuring the normal development of PTIs is the focus in the targeted intervention of PTIs. In this study, better nutritional status and growth and development status were determined in PTIs in the KMC group, demonstrating the excellent intervention effect of KMC on newborns under breastfeeding. In the study of Ramani M et al., we also found more significant improvements in growth and development of full-term infants with hypothermia under KMC intervention [23], which can also corroborate the results of this experiment. The main reasons for the difference in growth and development between groups, we speculate, may be the following: (1) early skin contact between mothers and infants can stimulate skin receptors into the cerebral cortex, reduce nerve tension, and promote the secretion of neonatal neurotransmitters, thus regulating the metabolism of growth hormone, thyroxine, and insulin levels. Besides, it can increase the catecholamine in newborns, promote the synthesis of glycogen, protein, and fat, and increase the intake of newborns [24]. (2) PTIs tend to lose heat easily due to thin subcutaneous fat and rich and sensitive blood vessels [25], while under the intervention of KMC, the amount of autonomic activity and the consumption of oxygen and heat are decreased. At the same time, skin contact can transfer the mother's temperature to the newborn and keep the body temperature constant, which is also conducive to physical growth. (3) Finally, the safe, stable, and warm environment created by KMC can stimulate the brain function development of neonates, which is conducive to the formation of synapses. Therefore, the implementation of KMC in breastfeeding can improve the growth and development of PTIs from multiple perspectives.

Among the organ dysfunctions of PTIs, abnormal immunological function and pulmonary function are the most common manifestations, and their abnormality is usually the key to the occurrence of major infectious diseases, respiratory arrest, and respiratory failure in PTIs [26]. In this study, we found effectively improved immunological function and pulmonary function of both groups after intervention, which highlighted the importance of breastfeeding for the growth and development of PTIs. More significant improvements were determined in the KMC group, indicating that the implementation of KMC in breastfeeding has a more effective promotion effect. The improvement, we speculate, may also be correlated with prone sleep of KMC in addition to the above speculations. As is known to all, due to the incomplete development of the respiratory system, PTIs may compress the lungs due to the heart, ribs, and other organs and tissues when they remain supine or side lying, reducing the compliance of the lungs and making it more difficult for the originally incomplete pulmonary function to operate [27]. By lying on the stomach, children can keep their lungs on top and their heart on the bottom, thereby reducing the compression area of lung tissue and helping the lungs to achieve the optimal level of expansion and compliance [28]. This state can not only more reliably maintain the normal operation of pulmonary function, but also enable the newborn to obtain a more stable respiratory cycle, contributing to a higher quality of sleep and rest. Similarly, when Aagaard et al. performed KMC on neonates in the intensive care unit, they found more effective improvements in pulmonary function [29]. Finally, the nursing satisfaction survey results of the two groups demonstrated that the implementation of KMC in breastfeeding has gained higher recognition of the delivery women, which once again confirmed its potential for clinical application.

While providing a good guarantee for the immunological function and pulmonary function of PTIs, the implementation of KMC under breastfeeding can effectively improve the efficiency of maternal breastfeeding and the growth and development of PTIs, which is worth promoting in clinical use. In the follow-up study, we will carry out a longer follow-up investigation on delivery women and PTIs in this study to analyze the long-term prognostic impact of KMC on PTIs. Second, it is necessary to increase the number of research subjects so as to obtain more representative results for clinical reference.

## Figures and Tables

**Figure 1:** The serum levels of PA, TRF, and ALB in the PTIs after KMC intervention. ^*∗*^*P* < 0.001 versus before intervention and ^#^*P* < 0.001 versus the control group.

**Figure 2:** The serum levels of Ig*A*, Ig*G*, Ig*M*, C_3_, and C_4_ in the PTIs after KMC intervention. ^*∗*^*P* < 0.001 versus before intervention and ^#^*P* < 0.001 versus the control group.

**Table 1:** Baseline data of delivery women and their PTIs.

	KMC (*n* = 46)	Control (*n* = 40)	*t* or *χ*^2^	*P*
Maternal age (year)	28.37 ± 3.16	28.90 ± 3.20	0.771	0.443
Sex of newborn, *n* (%)			0.086	0.769
Boy	25 (54.35%)	23 (57.50%)		
Girl	21 (45.65%)	17 (42.50%)		
Maternal BMI (kg/cm^2^)	28.19 ± 1.96	28.62 ± 1.15	1.217	0.227
Gestational age (week)	30.37 ± 1.78	30.63 ± 1.81	0.670	0.505
Weight at birth (g)	1742 ± 123	1723 ± 121		
Primiparity, *n* (%)			0.024	0.878
Yes	28 (60.87%)	25 (62.50%)		
No	18 (39.13%)	15 (37.50%)		
Nationality, *n* (%)			0.090	0.764
Han nationality	43 (53.48%)	38 (95.00%)		
Minority	3 (6.52%)	2 (5.00%)		

**Table 2:** KMC intervention benefits breastfeeding status of PTIs.

	KMC (*n* = 46)	Control (*n* = 40)	*t*	*P*
The time of first lactation (h)	39.14 ± 3.97	45.71 ± 5.43	6.46	<0.001
The time of first breastfeeding (h)	38.89 ± 4.16	49.68 ± 4.78	11.19	<0.001
The duration of first breastfeeding (min)	12.87 ± 2.46	6.08 ± 1.02	16.27	<0.001
LATCH scores	7.07 ± 0.98	6.25 ± 1.77	2.70	0.008

**Table 3:** KMC intervention benefits maternal psychological state after KMC intervention.

	Time point	KMC (*n* = 46)	Control (*n* = 40)
BSES score	Before intervention	49.17 ± 3.64	50.80 ± 3.53
	After intervention	93.72 ± 4.72^*∗*^^#^	71.90 ± 5.71^*∗*^
SAS score	Before intervention	57.13 ± 4.49	55.78 ± 4.64
	After intervention	30.72 ± 3.40^*∗*^^#^	48.40 ± 3.62^*∗*^
SDS score	Before intervention	57.98 ± 4.77	57.08 ± 3.80
	After intervention	31.67 ± 3.51^*∗*^^#^	48.33 ± 3.80^*∗*^

^*∗*^ *P* < 0.001 versus before intervention and ^#^*P* < 0.001 versus the control group.

**Table 4:** The growth status of PTIs after KMC intervention.

	KMC (*n* = 46)	Control (*n* = 40)	*t*	*P*
Weight gain (g/d)	4.29 ± 0.58	3.78 ± 0.42	4.61	<0.001
Body length gain (cm/week)	1.32 ± 0.14	0.93 ± 0.14	12.89	<0.001
Head circumference increase (cm/week)	1.30 ± 0.16	1.01 ± 0.13	9.14	<0.001
Upper arm circumference increase (cm/week)	0.62 ± 0.27	0.43 ± 0.19	3.72	<0.001

**Table 5:** KMC intervention benefits the pulmonary function of PTIs after KMC intervention.

	Time point	KMC (*n* = 46)	Control (*n* = 40)
VT (mL)	Before intervention	15.01 ± 4.18	15.85 ± 4.61
	After intervention	24.79 ± 4.91^*∗*^^#^	20.91 ± 2.75^*∗*^
VT/kg (mL)	Before intervention	5.22 ± 0.74	5.38 ± 0.81
	After intervention	7.74 ± 1.51^*∗*^^#^	6.43 ± 1.02^*∗*^
MV (L)	Before intervention	0.69 ± 0.08	0.68 ± 0.07
	After intervention	1.55 ± 0.16^*∗*^^#^	1.15 ± 0.08^*∗*^
MV/kg (L)	Before intervention	0.23 ± 0.06	0.24 ± 0.05
	After intervention	0.46 ± 0.08^*∗*^^#^	0.38 ± 0.07^*∗*^

^*∗*^ *P* < 0.001 versus before intervention and ^#^*P* < 0.001 versus the control group.

**Table 6:** Maternal satisfaction survey results.

	Very satisfied	Basically satisfied	Improvement needed	Dissatisfied
KMC (*n* = 46)	39 (84.78)	7 (15.22)	0 (0.0)	0 (0.0)
Control (*n* = 40)	21 (52.50)	14 (35.00)	3 (7.50)	2 (5.00)
*χ* ^2^	10.570	4.537	3.575	2.355
*P*	0.001	0.033	0.059	0.125

## Data Availability

The data supporting the findings of this study are included in this article.
